The article "Analysis of the Influencing Factors of Sentinel Lymph Node Metastasis in Breast Cancer" was retracted in 2023. Reasons: signs of a paper mill; compromised peer review; unreliable results or conclusions.

# Analysis of the Influencing Factors of Sentinel Lymph Node Metastasis in Breast Cancer

**DOI:** 10.1155/2022/5775971

**Published:** 2022-08-09

**Authors:** Wei Lyu, Yujuan Guo, Haiyan Peng, Nanyu Xie, Hongyi Gao

**Affiliations:** Department of Pathology, Guangdong Women and Children Hospital, Guangzhou 511400, China

## Abstract

**Objective:**

To analyze and discuss the influencing factors of sentinel lymph node metastasis in breast cancer.

**Methods:**

A total of 469 breast cancer patients admitted in the Department of Pathology of Guangdong Women and Children Hospital from October 2016 to December 2021 were retrospectively analyzed. The general information, immunohistochemical expression, tumor molecular subtype, tumor size, histological grade, pathological type, and tumor location were collected and the relationship with sentinel lymph node metastasis was analyzed.

**Results:**

For patients with different age, Ki-67 and Human epidermal growth factor receptor-2 (HER-2) immunohistochemical expression level (invasive cancer), molecular subtype (invasive cancer), tumor size, histological grade (invasive cancer) and pathological type. The results of multivariate logistic regression analysis showed that the age was less than or equal to 40 years; the molecular subtype was Luminal B and HER-2 overexpression (invasive cancer); tumor was larger; the histological grade (invasive cancer) was higher; the pathological type was invasive carcinoma, there were independent risk factors for sentinel lymph node metastasis in breast cancer. The sentinel lymph node metastasis rates of invasive lobular carcinoma, invasive micropapillary carcinoma, and metaplastic carcinoma (all met the criteria for squamous cell carcinoma and histological grade III) were higher than 50% in special invasive carcinomas.

**Conclusion:**

Age, expression level of Ki 67 and HER-2, molecular typing, tumor volume and histological grade are all high-risk factors related to sentinel lymph node metastasis of breast cancer. When one or more of the above factors are involved in an examination, pathologists should be more cautious in making a sentinel lymph node frozen diagnosis. By standardizing the sampling and increasing the number of frozen sections (slicing more frozen tissue layers), the section quality can be improved. This may be conducive to reducing the false negative rate and reducing the pain and risk of secondary surgery.

## 1. Introduction

Globally, breast cancer is the most common female malignancy, accounting for approximately one quarter of all cancers, and the incidence remains high [1, 2]. Compared with Europe and the United States, the incidence of the disease has increased in China, especially in rural areas [3–6]. However, due to advances in cancer screening and treatment, breast cancer mortality has declined significantly in recent years [7–9]. At present, the treatment of breast cancer mainly includes surgery, radiotherapy and chemotherapy, endocrine therapy, targeted therapy, and immunotherapy. Although the treatment methods are constantly enriched and the survival rate has improved, the associated adverse reactions still compromise the quality of life of patients. A number of studies have shown that the combination of traditional Chinese and Western medicine in the treatment of breast cancer can reduce the adverse reactions of radiotherapy and chemotherapy, enhance the body's immunity, effectively prevent the recurrence and metastasis of breast cancer, significantly improve the quality of life of patients, and prolong the survival time of patients. However, there is currently no unified standard for TCM syndrome types of breast cancer, and its application has not been popularized [10].

The article "Analysis of the Influencing Factors of Sentinel Lymph Node Metastasis in Breast Cancer" was retracted in 2023. Reasons: signs of a paper mill; compromised peer review; unreliable results or conclusions.

Originating from the study of penile cancer, the sentinel lymph node (Sentinel lymph node, SLN) refers to the lymph nodes that first metastasize to the tumor, which can be one or a group of lymph nodes. In sentinel lymph node biopsy (SLNB), the lymph nodes are marked with tracers, and after excision, a pathological examination is performed [11]. When the pathological result of SLNB is negative, dissection of the axillary lymph nodes may not need to be performed to avoid metastasis. It can reduce trauma and significantly improve the quality of life after surgery [12–14]. When the results are positive, axillary lymph node dissection may be necessary.

The pathological diagnosis of SLNB is performed by intraoperative frozen section examination of the sentinel lymph nodes. Due to the limitations of frozen tablets, even with standardized procedures, misdiagnosis still exists, especially for sentinel lymph node micrometastases [15]. Patients may bear the pain and risk of a second surgery. This study analyzed the influencing factors of sentinel lymph node metastasis in breast cancer patients. In the event that there are one or more high-risk factors, pathologists should be more cautious when making a sentinel lymph node frozen diagnosis to reduce the false-negative rate of pathology.

## 2. Methods and materials

### 2.1. Baseline Data

The data of the cases of breast cancer diagnosed by the Department of Pathology of Guangdong Women and Children Hospital from October 2016 to December 2021 were reviewed.

### 2.2. Inclusion Criteria

All punctured or minimally invasive surgeries were treated with immunohistochemical estrogen receptor (ER), progesterone receptor (PR), Ki-67, and human epidermal growth factor receptor-2 (HER-2). All cases underwent intraoperative sentinel lymph node frozen section examination after confirmation. All cases were primary breast tumors, and none of the patients received neoadjuvant therapy.

The article "Analysis of the Influencing Factors of Sentinel Lymph Node Metastasis in Breast Cancer" was retracted in 2023. Reasons: signs of a paper mill; compromised peer review; unreliable results or conclusions.

### 2.3. Data Collection Method

The patient's age, immunohistochemical expression, tumor molecular subtype, tumor size, histological grade, pathological type, tumor location, and other clinical and pathological data were queried and collected through the pathological diagnosis system and electronic medical record system. Four hundred and sixty-nine cases of standardized breast cancer were included.

### 2.4. Statistical Analysis

All data were processed by SPSS 19.0 software. According to the nature of the data and the purpose of the study, chi square analysis and multivariate logistic regression analysis were performed. *P* values<0.05 were deemed as significant.

## 3. Results

### 3.1. Sentinel Lymph Node Metastasis of Breast Cancer

A total of 469 cases of breast cancer were included, including 41 cases (8.74%) of breast carcinoma in situ, no cancer metastasis in sentinel lymph nodes (0.00%); There were 428 cases of breast invasive carcinoma (91.26%) and 139 cases of sentinel lymph node metastasis (32.48%).

### 3.2. Univariate Analysis of Sentinel Lymph Node Metastasis

The results indicated that there were significant differences in sentinel lymph node metastasis rates among breast cancer patients of different ages, Ki-67 and HER-2 immunohistochemical expression levels (invasive carcinoma), molecular subtypes (invasive carcinoma), tumor size, histological grade (invasive carcinoma) and pathological types (*P* < 0.05) as shown Table 1.

### 3.3. Multivariate Logistic Regression Analysis of Influencing Factors of Sentinel Lymph Node Metastasis

Using sentinel lymph node metastasis as a dependent variable, age, Ki-67 (IHC), HER-2 (IHC), molecular subtype, tumor size, histological grade, and pathological type as independent variables, multivariate logistic regression analysis was performed. See Table 2 for assignment of independent variables. The results indicated that age ≤40, molecular subtypes of luminal B and HER-2 overexpression (infiltrating carcinoma), the larger the tumor, the higher the histological grade (infiltrating carcinoma), and the pathological type of infiltrating carcinoma were independent risk factors for sentinel lymph node metastasis of breast cancer (*P* < 0.05). See Table 3.

### 3.4. Sentinel Lymph Node Metastasis of Special Invasive Carcinoma

The sentinel lymph node metastasis rate of invasive lobular carcinoma, invasive micropapillary carcinoma, and metaplastic carcinoma (all conform to squamous cell carcinoma, histological grade III) in special invasive carcinoma was higher than 50%. See Table 4.

The article "Analysis of the Influencing Factors of Sentinel Lymph Node Metastasis in Breast Cancer" was retracted in 2023. Reasons: signs of a paper mill; compromised peer review; unreliable results or conclusions.

## 4. Discussion

Sentinel lymph node metastasis is related to surgical method choice and prognosis [11, 12]. Intraoperative frozen section examination can determine the status of sentinel lymph nodes, but due to limitations, there is a false negative rate of about 10% [18]. If the associated high-risk factors are noted, better preparation for frozen collection and frozen section may reduce the false-negative rate of pathology.

This study suggested that when the patient was less than or equal to 40 years old, the immunohistochemical expression level of Ki-67 and HER-2 was higher (invasive cancer), the molecular subtype was Luminal B and HER-2 overexpression (invasive cancer), the tumor was larger, histological grade (invasive cancer) was higher, and the pathological type included invasive lobular carcinoma, invasive micropapillary carcinoma, metaplastic carcinoma. We should consider these to be high-risk factors for sentinel lymph node metastasis.

In this study, in the age ≤40 group, the sentinel lymph node metastasis rate was about 40.54%, and in the age>40 groups was about 27.59%. Patients aged less than or equal to 40 were defined as young breast cancer patients [16] and had more adverse prognostic factors compared with middle-aged and elderly patients, including larger lesions, poor differentiation, HER-2 overexpression, triple negative type and vascular invasion are more common, have higher histological grades, are more prone to lymph node metastases, and have more metastases [17, 18]. Presumably, young breast cancer patients have high levels of endogenous estrogen in the blood. They tend to develop rapidly after developing breast cancer, the disease is mostly in the advanced stage, and it is more likely to have axillary lymph node metastasis, blood or bone metastasis in the early stage [19]. In addition, young breast cancer patients are at reproductive age, their clinical symptoms are not typical, and the physiological hyperplasia and development of the breast make the tumor difficult to discover on their own. Together, the late treatment, the dense breast gland tissue, and the low sensitivity of B-ultrasound and mammography are also the influencing factors.

Ki-67 is a nuclear protein that is expressed in various stages of cell proliferation (G1, S, G2, M), but not in cell quiescence (G0). Therefore, Ki-67 can detect the proliferation activity of normal tissue and tumor tissue. The higher the Ki-67 index, the more aggressive the breast cancer and the worse the prognosis [18, 20]. HER-2 is a tyrosine kinase transmembrane protein involved in the regulation of multiple intracellular signaling pathways and is associated with breast cancer cell proliferation and apoptosis. HER-2 positive with obvious nuclear atypia, poor tumor differentiation, and high number of lymph node metastases, are associated with poor prognosis of patients [18, 21]. Our findings were similar to the above findings.

The article "Analysis of the Influencing Factors of Sentinel Lymph Node Metastasis in Breast Cancer" was retracted in 2023. Reasons: signs of a paper mill; compromised peer review; unreliable results or conclusions.

According to St Gallen [22], breast cancer is divided into four molecular subtypes, including ① luminal A: ER positive, HER-2 negative, Ki67 < 14%, or Ki67 at 14%–19% and PR>20%; ② luminal B: ER positive, HER-2 negative, Ki67 > 20%, or Ki67 at 14%–19% and PR negative or PR<20%, or ER positive, HER-2 positive; ③ HER-2 overexpression: ER negative, PR negative, and HER-2 positive; ④ triple negative: ER negative, PR negative, HER-2 negative. In this study, the molecular subtypes Luminal B and HER-2 overexpressed sentinel lymph node metastasis rates were higher (42.77% and 43.75%, respectively), compared with Luminal A (22.98%) and triple negative (18.87%). Similar to the findings of Wang Kanghan [23], this may be related to the higher expression levels of Ki67 or HER-2 in the molecular subtype Luminal B and HER-2 overexpression. Relevant studies [24, 25]showed that breast cancer tumor size was positively correlated with lymph node metastasis, which may be because the larger the tumor size, the more likely it is to have invasive cancer and the greater the possibility of invading vessels. Some patients received neoadjuvant therapy before surgery, which affected the actual size of the tumor and lymph node status, so these cases were excluded from this study. The results of this study showed that with the enlargement of the tumor, the rate of sentinel lymph node metastasis increased.

Breast cancer was histologically graded by assessing the degree of tubular and glandular differentiation, nuclear pleomorphism, and mitotic counts in invasive carcinomas. With these indicators, the histological grade of breast cancer is significantly correlated with the prognosis of patients [26, 27]. The severity of tumor differentiation, nuclear atypia, mitotic figures, and lymph node metastasis rates varies from grade I to grade III in histological grades. This study showed that the sentinel lymph node metastasis rate of breast cancer histological grade I was 6.45%, that of grade II was 37.05%, and that of grade III was 47.62%.

Invasive lobular carcinoma accounts for approximately 5–15 percent of invasive breast cancers, and studies showed that there were more lymph node metastases than nonspecialized invasive carcinomas [28]. This may be related to the loss of E-cadherin expression in invasive lobular carcinoma. E-cadherin is a cadherin, which can maintain intercellular adhesion and cell polarity. When the tumor tissue lacks or expresses low E-cadherin, it indicates aggressive [29]. Invasive micropapillary carcinoma accounts for approximately 3–8 percent of invasive breast cancers [30] and has a high rate of axillary lymph node metastasis [31]. Under electron microscopy, invasive micropapillary carcinoma cells have abnormally abundant filaments in the cytoplasm, which are highly mobile and invasive. In addition, cancer cells have been observed to contact the vascular endothelium through microvilli, which may be involved in tumor metastasis [32]. Metaplastic carcinomas are a group of tumors characterized by tumor epithelial differentiation to squamous and/or mesenchymal elements. Two cases of metaplastic carcinoma in this study all met the criteria for squamous cell carcinoma and histological grade III. Sentinel lymph node metastasis was observed in both cases.

The article "Analysis of the Influencing Factors of Sentinel Lymph Node Metastasis in Breast Cancer" was retracted in 2023. Reasons: signs of a paper mill; compromised peer review; unreliable results or conclusions.

There are still several limitations in this study. First, this study is a retrospective research analysis, and the retrospective study itself has certain defects; second, the sample size of this study is too small, it lacks representativeness, and the results might lack generalizability, which may bias the conclusion.

## 5. Conclusion

Age, expression level of Ki 67 and HER-2, molecular typing, tumor volume, and histological grade are all high-risk factors related to sentinel lymph node metastasis of breast cancer. When one or more of the above factors are involved in an examination, pathologists should be more cautious in making a sentinel lymph node frozen diagnosis. By standardizing the sampling and increasing the number of frozen sections (slicing more frozen tissue layers), the section quality can be improved. This may be conducive to reducing the false negative rate and reducing the pain and risk of secondary surgery.

## Figures and Tables

**Table 1:** Univariate analysis (*n* (%)).

Interfering factors	*n*	No metastasis	With metastasis	*χ2*	*P*
Age					
≤40	74	44 (59.46)	30 (40.54)	5.01	0.03
>40	395	286 (72.41)	109 (27.59)		
Ki-67					
≤30%	196	153 (78.06)	43 (21.94)	24.93	≤0.01
30%∼60%	114	76 (66.67)	38 (33.33)		
>60%+	118	60 (50.85)	58 (49.15)		
HER-2					
Negative	196	151 (77.04)	45 (22.96)	19.52	≤0.01
Unsure	172	109 (63.37)	63 (36.63)		
Positive	60	29 (48.33)	31 (51.67)		
Molecular subtype					
Luminal A	161	124 (77.02)	37 (22.98)	21.90	≤0.01
Luminal B	166	95 (57.23)	71 (42.77)		
HER-2expression	48	27 (56.25)	21 (43.75)		
Sanyin type	53	43 (81.13)	10 (18.87)		
Size of tumor					
≤2 cm	234	176 (75.21)	58 (24.79)	7.26	0.03
2∼5 cm	219	146 (66.67)	73 (33.33)		
>5 cm	16	8 (50.00)	8 (50.00)		
Histological grade					
I	93	87 (93.55)	6 (6.45)	39.90	≤0.01
II	251	158 (62.95)	93 (37.05)		
III	84	44 (52.38)	40 (47.62)		
Pathological type					
Carcinoma in situ	41	41 (100.00)	0 (0.00)	22.11	≤0.01
Nonspecific	369	238 (64.50)	131 (35.50)		
Specific	59	36 (61.02)	23 (38.98)		
Region					
Outer upper quadrant	201	136 (67.66)	65 (32.34)	6.41	0.17
Outer lower quadrant	77	58 (75.32)	19 (24.68)		
Inner upper quadrant	97	74 (76.29)	23 (23.71)		
Inner lower quadrant	36	27 (75.00)	9 (25.00)		
Posterior papilla	58	35 (60.34)	23 (39.66)		

Note. The pathological molecular subtypes and histological grades of breast cancer are only analyzed for the components of invasive breast cancer. Because no sentinel lymph node metastasis occurred in breast carcinoma in situ, in order to eliminate its interference, factors such as “Ki-67 (IHC),” HER-2 (IHC) “only analyzed cases of invasive breast cancer.

The article "Analysis of the Influencing Factors of Sentinel Lymph Node Metastasis in Breast Cancer" was retracted in 2023. Reasons: signs of a paper mill; compromised peer review; unreliable results or conclusions.

**Table 2:** Assignment of multivariate logistic regression analysis.

Factors	Evaluation
Age	≤40 = 1; >40 = 2
Ki-67 (IHC)	≤30% = 1; 30∼60% = 2; >60%+ = 3
HER-2 (IHC)	Negative = 1; Unsure = 2; Positive = 3
Molecular subtype	Luminal *A* = 1; luminal *B* = 2; HER-2+ = 3; sanyin type = 4
Size of tumor	≤2 cm = 1; 2∼5 cm = 2; >5 cm = 3
Histological grading	I = 1; II = 2; III = 3
Pathological type	Carcinoma in situ = 1; nonspecific = 2; special = 3

**Table 3:** Multivariate logistic regression analysis.

Influential factors	B	SE	Wald *χ*2	*P*	OR	95% CI
Age	0.760	0.227	11.256	0.001	2.139	(1.372, 3.336)
Ki-67 (IHC)	0.226	0.133	2.895	0.089	1.254	(0.966, 1.626)
HER-2 (IHC)	−0.052	0.132	0.156	0.693	0.949	(0.734, 1.229)
Molecular subtype	−0.290	0.099	8.624	0.003	0.748	(0.616, 0.908)
Tumor size	−0.554	0.140	15.724	≤0.001	0.575	(0.437, 0.756)
Histological grading	0.279	0.134	4.364	0.037	1.322	(1.017, 1.717)
Pathological type	0.332	0.134	6.117	0.013	1.394	(1.071, 1.814)

**Table 4:** Sentinel lymph node metastasis of special invasive carcinoma (*n* (%)).

Special invasive carcinoma	*n*	No metastasis	Metastasis
Invasive lobular carcinoma	10	3 (30.00)	7 (70.00)
Tubular carcinoma	5	5 (100.00)	0 (0.00)
Cribriform carcinoma	2	2 (100.00)	0 (0.00)
Mucinous carcinoma	20	19 (95.00)	1 (5.00)
Invasive micropapillary carcinoma	15	4 (26.67)	11 (73.33)
Carcinoma with apocrine differentiation	5	3 (60.00)	2 (40.00)
Metaplastic carcinoma	2	0 (0.00)	2 (100.00)

Note: the tumors in the table are sorted according to the catalog of breast tumors.

## Data Availability

No data were used to support this study.
